This article has been retracted.

# Analysis of Relevant Factors Affecting the Pregnancy Rate of Frozen-Thawed Embryo Transfer Cycle

**DOI:** 10.1155/2022/2842278

**Published:** 2022-05-18

**Authors:** Ning Liu, Yuhong Wang, Jing Lu, Xihui Zhang, Yunjing Zhang, Haijun Zhao, Yijiao Zhang, Wenliang Chang

**Affiliations:** Department of Reproductive Medicine, Handan Central Hospital, Handan 056000, Hebei Province, China

## Abstract

**Objective:**

The aim of this study is to explore the relevant factors affecting the pregnancy rate of frozen-thawed embryo transfer cycle.

**Methods:**

The clinical data of 931 patients who underwent artificial cycle preparation for endometrial FET from April 2017 to November 2020 in the reproductive center of our hospital were retrospectively analyzed.

**Results:**

According to the pregnancy situation, the patients were divided into 450 cases of pregnancy and 481 cases of biochemical pregnancy. The univariate analysis of FET biochemical pregnancy showed that there were statistically significant differences between pregnancy and biochemical pregnancy in terms of years of infertility, age, endometrial thickness, P level, E2/P, and the number of high-quality embryos (*P* < 0.05). Multivariate analysis of pregnancy showed that age <30 years was a protective factor for biochemical pregnancy and endometrial thickness <8 mm and E2/P < 0.3 were risk factors (*P* < 0.05).

**Conclusion:**

The regulation of endometrial thickness and E2/P serves as the key of treatment for patients undergoing FET using artificial cycle preparation for endometrial transfer, and it contributes to improve the pregnancy rate; also, the patient's age is an important indicator influencing the pregnancy rate.

## 1. Introduction

Embryonic implantation is predominantly associated with the quality of embryos, the receptivity of the endometrium, and whether the embryonic development is synchronized with the endometrium [1, 2]. With the constant advancements of the level of assisted reproductive technology, high-quality embryo obtainment is no longer a clinical problem. Nevertheless, the pregnancy rate of patients remains less than satisfactory, mainly due to poor endometrial receptivity [3, 4]. Since the success of frozen-thawed human embryo transfer in Australia in 1983, frozen-thawed embryo transfer (FET) technology has been widely used in the field of human Assisted Reproductive Technology (ART) due to its high cumulative pregnancy rate. The methods of preparing the intima mainly include a natural cycle and an artificial cycle. The artificial cycle is a process of simulating the action of the natural ovulation cycle hormone changes on the endometrium, thereby affecting the receptivity of the endometrium. Numerous studies have favored the use of natural cycles for endometrial preparation, concerning the safety of drugs for endometrial preparation and pregnancy rates [5, 6]. However, it is worth noting that the artificial cycle can choose the best time for embryo transfer, with a low cancellation rate. More importantly, its pregnancy rate is equivalent to, or even higher than, the natural cycle. In recent years, artificial cycle preparation has received more and more attention, but the incidence of biochemical pregnancy in some centers is still high, or even significantly increased [7]. At present, there are few reports on the pregnancy rate and biochemical pregnancy rate of frozen-thawed embryo transfer at home and abroad. This study explored the influencing factors of the pregnancy rate of frozen-thawed embryo transfer in order to reduce the biochemical pregnancy rate of FET. The innovation of this study lies in the collection and comparison of the two groups of data, obtaining the relevant risk factors, and using it as a guide in the clinical application. To this end, the pregnancy outcomes of 931 frozen-thawed embryo transfer cycles were compared and analyzed in the present study, and the related factors affecting the biochemical pregnancy of the frozen-thawed embryo transfer cycles were investigated.

In this section, we present the introduction about the paper, the next part involves study data and methods, followed by the results of our study, and finally, the discussion targeting the results is presented, and at last, the conclusion is drawn.

## 2. Study Design and Participants

### 2.1. Participants

The clinical data of 931 patients who underwent FET in the endometrium prepared by the artificial cycle from April 2017 to November 2020 in the reproductive center of our hospital were retrospectively analyzed. The age range was 21–48 years; the infertility period was 1–20 years. Those who did not ovulate naturally due to various reasons or those with infertility (including age of less than 48, no abnormal uterine cavity morphology in hysteroscopy, tubal obstruction, hydrosalpinx, ovulation disorders, male causes, etc.) were eligible to participate in the study. Whereas, those with repeated endometrial thickness of about 7 mm on the day of intramuscular injection of human chorionic gonadotropin (hCG) or luteal support and the presence of hydrosalpinx, scar diverticulum, endometriosis, adenomyosis, uterine fibroids surgical history, chromosomal polymorphism, thyroid function disease, autoimmune disease, polycystic ovary syndrome, uterine malformation, intrauterine adhesions, and endometrial polyps were excluded from the study. The protocol was approved by the ethics committee of Handan Central Hospital (9779-0279). All subjects gave written informed consent in accordance with the Declaration of Helsinki.

### 2.2. Methods

① Superovulation procedure: All patients who underwent *in vitro* fertilization-embryo transfer (including *in vitro* fertilization (IVF) or intracytoplasmic sperm injection (ICSI)) were treated with a gonadotropin-releasing hormone receptor agonist (GnRH- a, Biolab: M00440) or gonadotropin-releasing hormone receptor antagonist (GnRH-ant, Biolab: M00441) to down the regulation and gonadotropin to promote follicle growth; when there are 2 follicles with diameter ≥18 mm or more than 3 follicles with diameter ≥17 mm, hCG (Dabitat, 0.1 mg/piece, Ferring, Denmark) 5000–10000 U/L was given, and egg retrieval was performed after 34–36 h. According to the quality of sperm, IVF or ICSI was used for fertilization, and the embryos were graded according to morphology. The cells with a uniform size, complete zona pellucida, and less cell debris are high-quality embryos. The high-quality embryos were vitrified and frozen, and the embryos were recovered on the day of embryo transfer. ② Artificial cycle preparation of the endometrial procedure: artificial cycle was used to prepare the endometrium; for patients with an irregular menstrual cycle, anovulation, and poor endometrial growth, estradiol valerate (Bayer Healthcare Co., Ltd. Guangzhou Branch) 2-6 mg/d was orally administered on the 2–3 rd day of menstruation according to the individual's previous endometrial condition and menstrual history. The levels of estradiol (E2), progesterone (P), and luteinizing hormone (LH) were detected on the 9th to 12th day of menstruation, and B-scan ultrasonography was performed to monitor the endometrium, and the serum E2 and *P* levels, E2/P and endometrial thickness, morphology were recorded. The dose of valeric acid E2 was increased for patients with a poor endometrial growth, and E2 was given via vagina. Finally, the endometrial and hormone levels were monitored; if the thickness of the endometrium was acceptable, it was classified as type AB (40–60 mg/d of progesterone was injected on the second day after injection of hCG5000-10000 U if transforming the endometrium was necessary (produced by Zhejiang Xianju Pharmaceutical Co., Ltd and the embryo transfer was performed after 3-day continuous intramuscular injection of progestin or blastocyst transfer on the 5th and 6th day.

### 2.3. Outcomes

①Determination of serum E2 and P levels and calculation of E2/P: 5 ml of fasting venous blood was collected from 8 : 00–9:00 on the day of hCG injection, serum was separated, serum E2 and P levels were detected by electrochemiluminescence, and E2/P was calculated. ②Embryos thawing indicators and judgment of pregnancy: the number of embryos after freezing and thawing was recorded, and the number of high-quality embryos transferred (according to the standard of high-quality embryos with number of cells >4 and fragments ≤25%) was documented; embryo blastomeres exceeding 50% of the blastomeres before freezing and thawing was considered to survive, and all blastomeres intact without damage were intact viable embryos, and high-quality embryos were selected for transfer. 14 days after embryo transfer, blood hCG >10 U/L was considered as biochemical pregnancy, and the luteal support was continued; 30 days after embryo transfer, vaginal B-ultrasonography was performed, and it was clinical pregnancy if the gestational sac and the original cardiac tube beat were seen in the uterus, and luteal support therapy was continued till 12 weeks of pregnancy. ③ Pregnancy rate: the number of pregnant patients ÷ the total number of cases × 100% = pregnancy rate.

### 2.4. Statistical Analysis

SPSS 21.0 statistical software was used to analyze the data, the count data are expressed as *n* (%), and the comparison between groups was performed by the X^2^ test; the FET biochemical pregnancy rate was analyzed by multivariate logistic regression. *P* < 0.05 was considered statistically significant.

## 3. Results

### 3.1. Univariate Analysis of Factors Influencing FET Biochemical Pregnancy

According to the pregnancy situation, the patients were divided into 450 cases of pregnancy and 481 cases of biochemical pregnancy. Infertility years, age, endometrial thickness, P level, E2/P, and the number of high-quality embryos were correlated with a clinical pregnancy outcome and pregnancy rate, and the difference was statistically significant (*P* < 0.05). See Table 1.

### 3.2. Multivariate Analysis of Factors Affecting FET Biochemical Pregnancy

According to univariate analysis, age, infertility years, endometrial thickness, *P* level, E2/P, and the number of high-quality embryos were used as independent variables, and biochemical pregnancy was used as a dependent variable for multivariate analysis. Multivariate logistic regression analysis showed that age < 30 is a protective factor for biochemical pregnancy, and endometrial thickness <8 mm and E2/*P* < 0.03 are risk factors (*P* < 0.05), as shown in Table 2.

## 4. Discussion

Recently, the low implantation rate of transferred embryos remains a major challenge [7, 8]. Some studies believe that the cause for the failure of embryo implantation is mainly due to the adverse effect of supraphysiological doses of hormones that stimulate ovulation on endometrial receptivity, resulting in the early opening of the “implantation window”. On the other hand, 10%–20% of patients have low levels of hormones, which can cause the endometrium to develop out of sync with the embryo [9–12].

To our knowledge, age is an important factor affecting female fertility, and the quality and quantity of a woman's eggs decline with age after puberty. In the use of assisted reproductive technology, age is the key to determine the pregnancy rate, since it is related to embryo quality. Studies argued that there is no significant difference in the pregnancy rate at the same age in the FET cycle of the natural cycle and the artificial cycle. Interestingly, this study compared the difference in pregnancy rates between patients <30 years and ≥30 years and found that the pregnancy rate was lower in patients ≥30 years. Additionally, regression analysis also showed that age was a related factor of pregnancy rate and believed that the impact of age on FET pregnancy rate was attributed to the fact that younger embryos exhibit better quality.

Some studies have analyzed the egg donation cycles of the same age group, and there is no significant difference in the pregnancy rate of recipients in different age groups, indicating that the effect of age on the successful clinical pregnancy of assisted reproductive technology is still determined by the quality of the embryo and is not related to the endometrial preparation program [13, 14]. In addition to embryo quality, the related factors of embryo implantation are endometrial receptivity. Endometrial receptivity refers to the ability of the endometrium to accept embryo positioning, adhesion, implantation, etc. The shape, thickness, subendometrial blood flow, and hormone receptor factors on the endometrium, all play a role in the endometrium receptivity and synchrony between the embryo and endometrium [15, 16]. At present, most studies have shown that the thickness of the endometrium on the day of endometrial transformation is related to the clinical pregnancy rate of FET, and the clinical pregnancy rate is higher when the thickness of the endometrium is within a certain range. Some researchers divided the endometrial thickness on the transition day of FET cycle into 7–12 mm group, >12 mm group, and ≤7 mm group, and found that the clinical pregnancy rate of the group with endometrial thickness ≤7 mm on the transition day was the lowest through a comparative study. This present study compared the clinical pregnancy rate of patients with different endometrial thickness (<8 mm, 8–10 mm, and ≥10 mm). The results showed that the clinical pregnancy rate of patients with different endometrial thicknesses was statistically different. Also, multivariate logistic regression analysis showed that endometrial thickness is a key factor affecting the pregnancy rate and pregnancy outcome of FET. Thus, when FET is performed, monitoring the endometrial thickness is of considerable clinical significance for patients with FET pregnancy [17].

In addition to a variety of cytokines and growth factors involved in regulating endometrial receptivity, E2 and P play a leading role in the process of embryo implantation. Many scholars believe that the establishment of endometrial receptivity requires an appropriate ratio of E2 and P, and the changes in endometrial receptivity can be monitored by adjusting E2/P to determine the time of embryo transfer and increase the probability of pregnancy [18–21]. Regarding the mechanism by which E2 and P act on the endometrium, we assumed that they may play a role by acting on the pinocytosis of the endometrium: on the one hand, P regulates the growth of pinocytosis, and on the other hand, E2 has a restrictive effect on it. Song et al. pointed out that E2/P is closely related to the pregnancy rate using logistic regression analysis. According to our study results, E2/P was significantly correlated with the clinical pregnancy rate of patients. Further logistic regression analysis found that E2/P was an important factor affecting pregnancy outcomes. In light of this, it is necessary to closely monitor and regulate the serum E2/P of patients during FET, which is beneficial to improve the probability of pregnancy.

## 5. Conclusion

The regulation of endometrial thickness and E2/P serves as the key of treatment for patients undergoing FET using artificial cycle preparation for endometrial transfer, which improves the pregnancy rate; the patient's age is an important indicator influencing the pregnancy rate. The limitation of the study should be outlined. There is no further study on the early detection and judgment of biochemical pregnancy patients with related drug interventions. In the future, trials with larger study participants will be conducted toward this direction.

## Figures and Tables

**Table 1:** Univariate analysis of factors influencing FET biochemical pregnancy [*n* (%)].

	*n*	Pregnancy (*n* = 450)	Nonpregnancy (*n* = 481)	x^2^	*P*
Cause of infertility				1.084	0.582

Female-side cause	745	361	384		

Male-side cause	160	79	81		

Other causes	26	10	16		

Age (year)				27.205	＜0.01
＜30	544	253	291		
≥30	387	114	273		

Infertility years (years)				5.256	0.022
≤3	678	258	420		
＞3	253	117	136		

Ovulation induction medication				1.945	0.163
CnRH-a	891	435	456		
CnRH-ant	40	15	25		

Fertilization method				3.777	0.052
IVF	757	377	380		
ICSI	174	73	101		

Endometrial thickness(mm)				7.412	0.025
＜8	224	95	129		
8–10	653	334	319		
＞10	54	21	33		

*E*_2_ (pg/ml)				5.378	0.068
＜200	422	221	201		
200–700	395	175	220		
＞700	114	54	60		

*P* (pg/ml)				7.110	0.029
＜0.3	345	148	197		
0.3–0.7	439	223	216		
＞0.7	147	79	68		

*E*_2_/*P*				13.143	0.001
＜0.3	174	87	87		
0.3–0.7	310	173	137		
≥0.7	447	190	257		

Number of high-quality embryos (*n*)				63.184	＜0.001
1	803	308	495		
≥2	128	97	31		

GnRH-a: gonadotropin-releasing hormone receptor agonist; GnRH-ant: gonadotropin-releasing hormone receptor antagonist; E2: estradiol; and P: progesterone.

**Table 2:** Multivariate analysis of factors influencing FET biochemical pregnancy.

Variable	*β*	Se	Wald	*P*	OR (95%CI)
Age	0.129	0.045	2.214	0.042	0.196 (0.068, 0.561)
Infertility years	0.321	0.032	2.456	0.365	0.523 (0.245, 0.756)
Endometrial thickness	0.384	0.106	13.242	0.000	1.468 (1.190, 1.806)
*P* Level	0.235	0.221	12.355	0.245	1.222 (1.054, 1.635)
*E*_2_/*P*	0.197	0.087	5.108	0.024	1.218 (1.027, 1.445)
Number of high-quality embryos	0.214	0.024	6.354	0.214	1.011 (0.987, 1.674)

Assignment: age is < 30 years = 0, ≥30 years = 1; infertility years are ≤ 3 years = 0, >3 = 1; endometrial thickness is < 8 mm = 1, 8–10 mm = 2, >10 mm = 3; *Pvalue* is < 0.3 pg/ml = 1, 0.3–0.7 pg/ml = 2, >0.7 pg/ml = 3; E2/*Pvalue* is < 0.3 = 1, 0.3–0.7 = 2, ＞0.7 = 3; the number of high-quality embryos is ≥2 = 0, 1 high-quality embryo = 1.

## Data Availability

The datasets used during the present study are available from the corresponding author upon reasonable request.
